This article has been retracted.

# Design and Optimization of Urinary Real-Time Nursing Model Based on Medical Internet of Things

**DOI:** 10.1155/2022/7067856

**Published:** 2022-04-20

**Authors:** Wei Hao, Xiujun Hao, Chao Yang

**Affiliations:** ^1^School of Chengde Medical University, Tangshan 063000, Hebei, China; ^2^School of North China University, Tangshan 063000, Hebei, China

## Abstract

The medical Internet of Things (IoTs) can bind intelligent sensing devices with urinary nursing recipients and integrate information into various hospital information systems through network communication, so as to realize the intelligent perception, data collection, remote monitoring, information sharing, and other functions of urinary real-time nursing recipients. The urinary real-time nursing model can complete the expansion of hospital information system data to the bedside and the instant exchange of terminal data with the system through the medical IoTs and wireless local area network. Based on the summary and analysis of previous research results, this paper expounds on the research status and significance of the urinary real-time nursing model, elaborates on the development background, current status, and future challenges of medical IoTs, introduces the methods and principles of medical IoTs level evaluation system and transformation rules-based optimization algorithm, conducts urinary real-time nursing model design based on medical IoTs, analyzes model hardware design based on medical IoTs, performs model software design based on medical IoTs, proposes the urinary real-time nursing model optimization based on medical IoTs, explores the front-end function optimization of the urinary real-time nursing, implements the system program optimization of the urinary real-time nursing, discusses the hierarchical architecture of the urinary real-time nursing model, and finally carries out the role function analysis of the medical IoTs in the urinary real-time nursing model. The study results show that the urinary real-time nursing model based on medical IoTs can accurately and efficiently identify, manage, and integrate clinical nursing procedures and data such as patients, diagnoses, drugs, and can optimize nursing workflow, strengthen quality control, and improve nursing efficiency and provide patients with more convenient nursing services. The research results of this paper provide a reference for further research on the design and optimization of urinary real-time nursing model based on medical IoTs.

## 1. Introduction

The medical Internet of things is a new application of the Internet in the medical industry, including the Internet as the carrier and technical means of health education, medical information query, electronic health records, disease risk assessment, online disease consultation, electronic prescription, remote consultation, and remote treatment and rehabilitation and other forms of health medical services. Internet medical treatment represents a new development direction in the medical industry and is conducive to solving the contradiction between the imbalance of medical resources in China and people's increasing demand for health and medical treatment. It is a medical development model actively guided and supported by the Ministry of Health.

Urinary real-time nursing model based on medical Internet of Things (IoTs) mainly aims at nurses' daily management of urinary disease patients' nursing work, realizes the informatization and standardization of nursing work, and ensures the smooth progress of nurses' mobile nursing work for patients [1]. According to the patient information and medication information or blood information collected by the handheld device, the real-time nursing model can accurately check the patient's information during the infusion process, the oral medication process, the blood sample collection process, and the vital signs input process [2]. It can send reminders to change the doctor's order and can also avoid repeated dispensing to ensure the safety of the patient's medication and to ensure the safety of the patient's life. The medical IoTs technology is displayed on the page after data conversion, and the value is stored in the corresponding database table. The model will also automatically summarize the qualification rates of all levels and various quality control indicators, reducing the links and time for quality control records at all levels and statistical quality control compliance rates. It has the functions of the most popular database development software at present, and the model adopts the international standard database when accessing the database [3]. For example, nurses are no longer limited to nurse stations and can freely read the patient's personal, hospitalization, and other diagnosis and treatment information in real time in the patient's ward or any other place in the hospital and can view real-time medical advice, physical signs, and other diagnosis and treatment information [4].

The urinary system is composed of kidneys, ureters, bladder, urethra, and related blood vessels and nerves. Its main function is to generate urine, excrete metabolites, regulate water, electrolyte, and acid-base balance, and maintain the stability of the body's internal environment. Details of general nursing in urology: except for special patients, patients should be encouraged to drink more water; routine urine collection should be kept, and midsection urine culture should be properly done. If there is a urinary tract infection, the operation should be postponed. Pay attention to observe possible reactions, such as anuria, urinary retention, dysuria, hematuria, chills, and fever. If there is an indwelling catheter (or ostomy tube), it should be properly fixed and kept unobstructed, and the drainage should be observed frequently. The color, quality, and quantity of the liquid should be rinsed regularly according to the doctor's instructions, and the drainage bottle (or drainage bag) should be replaced once a day; patients with urine leakage should keep the bed sheets dry to avoid pressure sores; pay attention to the patient's urination.

The continuous development of Internet technology has enabled the medical industry to enter the digital age, and Internet technology has also begun to be used in clinical nursing, which has simplified and upgraded the work of medical staff. With the continuous development of the Internet, the medical IoTs have begun to enter the clinical urinary real-time nursing system, which has brought more convenience to the hospital staff [5]. The hospital's information system can be connected to and transformed with the clinical information system, making the hospital's work process more convenient, improving the overall work efficiency of the hospital, and making the hospital's service satisfaction better [6]. The urinary real-time nursing model based on medical IoTs is applied to many aspects such as hospital staff management, item management, medical nursing, environmental monitoring, and information management, optimizing the urinary real-time nursing model and improving the overall efficiency of the hospital. The nursing model based on medical IoTs can optimize the nursing workflow, strengthen the quality control of the links, improve the efficiency of nursing work, and provide patients with more convenient nursing services [7]. The medical IoTs provide transparent data through the communication layer and, at the same time, obtain the patient's physiological information through the perception layer and can reflect the information to the nurses through the network layer [8].

Based on the summary and analysis of previous research results, this paper proposes the urinary real-time nursing model optimization based on medical IoTs, explores the front-end function optimization of the urinary real-time nursing, implements the system program optimization of the urinary real-time nursing, discusses the hierarchical architecture of the urinary real-time nursing model, and finally carries out the role function analysis of the medical IoTs in the urinary real-time nursing model. The detailed chapters are arranged as follows: Section 2 introduces the methods and principles of medical IoTs level evaluation system and transformation rules-based optimization algorithm; Section 3 conducts urinary real-time nursing model design based on medical IoTs; Section 4 proposes the urinary real-time nursing model optimization based on medical IoTs; Section 5 discusses the hierarchical architecture of the urinary real-time nursing model and carries out the role function analysis of the medical IoTs; Section 6 is the conclusion. The design process is to determine the design content, analyze design methods and principles, design scheme, design model, and find the shortcomings of the model of optimization, then test the optimized model, and finally draw a conclusion.

The innovation of this article is mainly combined with the traditional urinary nursing model, the design, and optimization, at the same time to test that the model analysis, consistency evaluation, and conclusion have credibility.

## 2. Methods and Principles

### 2.1. Level Evaluation System of Medical IoTs

This study uses the coordination coefficient *A*_*i*_ to test the consistency of the recognition of the index by experts. The value of the coordination coefficient is in the range of [0, 1]. The larger *A*_*i*_ indicates, the better the degree of coordination between experts. That is, the experts participating in the research have a higher evaluation consistency for each indicator, and when the *A*_*i*_ value is less than 0.5, it indicates that the coordination of a certain indicator is not good. Coordination coefficient can be used to test expert identification consistency. If the experts are consistent with each index, the evaluation results of experts on the medical Internet of Things model or scheme design level are more obvious, and vice versa. The calculation formula of the coordination coefficient *A*_*i*_ is as follows:

(1) $$\begin{array}{c} A_{i}=\frac{a_{j}\left(i\right)-b_{j}\left(i\right)}{c_{j}\left(i\right)-d_{j}\left(i\right)}, \end{array}$$

where *a*_*j*_ is the total evaluation level assigned to the *j*-th index; *b*_*j*_ is the total number of experts assigned to the *j*-th index; *c*_*j*_ is the standard deviation of the recognition of index *j*; *d*_*j*_ is the average of the recognition of index *j*; *i* is the index total.

Due to the beating of the heart, blood will periodically rush into the arteries to cause continuous changes in blood pressure. During this process, the blood vessel wall will also be slightly deformed. At this time, the changes in the inner diameter of the arterial wall and the thickness of the arterial wall can be ignored:

(2) $$\begin{array}{c} B_{i}=\frac{{\left|e\right|}^{-n}f_{i}\left(x\right)\cdot f_{i}\left(y\right)}{\langle g_{i}\left(x\right),g_{i}\left(x\right)\rangle }, \end{array}$$

where *e* is the pulse wave propagation distance; *n* is the pulse wave transit time; *f*_*i*_ is the elastic modulus when the pressure is zero; *x* is the blood pressure; *y* is the thickness of the blood vessel wall; *g*_*i*_*g*_*i*_ (*x*) is the fluid density; (*y*) is the inner diameter of the elastic tube; *f*_*i*_(*x*) is the pressure change; *f*_*i*_(*y*) is the fluid height change.

The system measures the patient's pulse, blood pressure, and body temperature information for a certain period of time. The pulse, blood pressure, and body temperature are set as feature vectors, which are represented by (*h*, *k*, *l*). In the three-dimensional number axis, these points will be expanded into a point set and the distance *C*_*i*_ of each point in the space is calculated as follows:

(3) $$\begin{array}{c} C_{i}=\frac{1}{p}\cdot \frac{{\left[h^{m}\left(i\right)-k^{m}\left(i\right)\right]}^{+}}{{\left[l^{o}\left(i\right)-k^{o}\left(i\right)\right]}^{+}}, \end{array}$$

where *m* is the *j*-dimensional coordinate value of the *i*-th feature point; *o* is the *j*-dimensional coordinate value of the *i*-th cluster point; *p* is the parameter value specified by the system, which is affected by the number of measurement data points in the time period, and there is a proportional relationship between them.

On the one hand, the urinary real-time nursing model is executed through the medical order collected by the medical IoTs, and the patient's physical sign information is updated in real time and uploaded to the data center to ensure timeliness and accuracy of information collection. On the other hand, the test result information collected by the model and the doctor's order information stored in the doctor's workstation are also concentrated in the data center; nurses can directly call the data center data through the mobile medical nursing system client to complete vital sign data query and test data query notification and many other operations [9]. The urinary real-time nursing model contains the business logic of the application, encapsulates the data needed to complete the business and the operations on the data, is the place for data processing and calculation, and reflects the state of the application. The real-time nursing model accepts the data requested by the view and returns the processing result. A model can provide data for multiple views at the same time, so the code used for the model can be reused by multiple views only once, which reduces code duplication and improves code reusability. The front controller dispatches requests to the handler and performs view resolution. It forwards it to a specific controller according to the user's request, and then the controller is responsible for processing the specific request and returning the model and view objects and the dispatcher parses the model and view.

### 2.2. Optimization Algorithm Based on Transformation Rules

According to the fusion clustering results of the urinary real-time nursing pipeline fault samples, the statistical time series analysis is performed, and the medical IoTs will extract the high-order spectral feature quantity of the urinary real-time nursing pipeline fault information. Higher-order spectral eigenvarieties refer to the statistics of order greater than second order, mainly including higher moments, higher-order cumulants, and higher-order cumulant spectrum (higher-order spectrum), which is an emerging new discipline. It can be used to identify noncausal, nonminimal phase systems or reconstruct nonminimal phase signals, extract various information caused by Gaussian deviation and nonlinearity in inspection and characterization signals, and identify nonlinear systems. Combining high-order statistical feature quantities and Atlas analysis methods, the sample fusion feature equation for adaptive equalization control of urinary real-time nursing pipeline operation failure is obtained as follows:

(4) $$\begin{array}{c} D_{i}=\frac{{\left(s\left\|r_{i}\right\|\right)}^{t}e^{-s\left\|r_{i}\right\|}}{q!}, \end{array}$$

where *D*_*i*_ is the output voltage vector distribution factor; *q* is the discrete number of faults in the urinary real-time nursing pipeline; *s* is the open-circuit control weight of the switch tube; *r*_*j*_ is the characteristic distribution of the faults in the urinary real-time nursing pipeline; *t* is the optimized value of power and energy.

Considering the above factors will help improve the enthusiasm and quality of nursing work. The two factors of nursing preference and tacit degree are soft constraints. In order not to reduce the chance of obtaining a feasible solution, they will be transformed into the objective function; therefore, the extended nursing scheduling problem model is as follows:

(5) $$\begin{array}{c} E_{i}=\overset{n}{\underset{i=1}{\sum }}D_{i}\left(x\right)=\overset{n}{\underset{i=1}{\sum }}D_{i}\left({\text{ud}}_{i}^{n}+{\text{vd}}_{i}^{n+1}+{\text{wd}}_{i}^{n+2}\right), \end{array}$$

where *u*, *v*, and *w* are the weight coefficients of nursing salary cost, preference, and tacit degree, and their values are assigned constants by the hospital according to the actual situation and can be required to satisfy *u*+ *v* +*w* = 1, *u*, *v*, *w* ∈[0, 1].

The general algorithm judges whether to accept the new solution, which only needs to judge whether the new solution meets the constraints and improves the objective function value. The importance sampling method is introduced in the simulated annealing algorithm, that is, to accept the new criterion with a certain probability. The commonly used acceptance criterion is as follows:

(6) $$\begin{array}{c} H_{i}=\left\{\begin{array}{c} \left(1-\frac{1}{I_{i}}\right)J_{i}\left(z-1\right)+\frac{1}{I_{i}}K_{i}\left(z-1\right),z\leq z_{i},\\ \left(1-\frac{1}{I_{i}}\right)J_{i}\left(z-1\right),z>z_{i}, \end{array}\right. \end{array}$$

where *I*_*i*_ is the model parameter; *J*_*i*_ is the difference of the objective function between the new solution and the current solution or the difference of the objective function between the current solution and the new solution; *K*_*i*_ is the random variable of the current solution; *z* is a discrete finite state space; *z*_*i*_ is the weighting factor of the optimization performance index.

Two basic rules are designed in the improvement phase of the urinary real-time nursing model based on medical IoTs: replacement rules and swap rules. The main steps are as follows: evaluate all nurses in the current model one by one; if the total number of nurses' work shifts is greater than the prescribed lower limit, use the replacement rule adjustment model; otherwise, if it is equal to the prescribed lower limit, use the swap rule adjustment model. Based on these two rules in such a rotation, the urinary real-time nursing model uses a descending algorithm to improve the current model until the model can no longer be improved or reaches the set number of iterations [10]. If the penalty value is zero, it is indicated as a feasible model, and the feasibility step of the model is terminated; otherwise, if the implementation of the above two rules, in turn, can no longer improve the current model, a random nurse from each level is selected, and the initial model assigns shifts to it and then repeats all the above operations until a feasible solution is found. This method can not only reduce the number of nurses assigned in shifts, but also tends to reduce nurses whose ability levels exceed the work level, which helps to balance the workload of nurses. Therefore, the nurse-reduction rules ensure that the current model is improved while taking into account the principle of balancing workload and talents.

## 3. Urinary Real-Time Nursing Model Design Based on Medical IoTs

### 3.1. Model Hardware Design Based on Medical IoTs

The urinary real-time nursing model based on medical IoTs is divided into the presentation layer, the application layer, and the data layer. The presentation layer is located on the user side, and the user side does not need to download the corresponding software and only needs to use the browser to realize the interaction with the server. Through the application layer, the information interaction between the presentation layer and the data layer can be realized, the request sent by the user can be received, and the data layer can be processed with business logic according to the content of the request. The data layer is the database server, which is responsible for direct interaction with the database, responding to requests from the application layer, and feeding back data to the application layer. After the buffer recognizes the data frame and receives the correct data frame, the software system needs to analyze the data frame and separate the data value contained in the data field and perform operations such as data type conversion. The medical IoTs is displayed on the page after data conversion, and the value is stored in the corresponding database table. By clicking the information management button, all bed information in the department can be displayed.  Figure 1 shows the hardware design of urinary real-time nursing model based on the medical IoTs.

The urinary real-time nursing model can make all parts cooperate with each other to complete data collection, reception, analysis, processing, post-release, and storage. This is the central hub of the medical IoTs information sharing platform and the exchange of hospitals and patients' diagnosis and treatment information. The urinary real-time nursing model is an intelligent management system suitable for hospital infusion, which is developed based on the IoTs technology, sensor technology, and database technology. After the nursing terminal analyzes and processes the patient's nursing progress in the form of data, it is transmitted to the intelligent infusion monitoring system in real time via the wireless network, and the system automatically calculates the remaining time for the completion of the infusion according to the infusion flow rate. During the nursing quality control inspection, the urinary real-time nursing model can directly input the problems found or click the problem option to generate input information. The model will also automatically summarize the qualification rates of all levels and various quality control indicators, reducing the links and time for quality control records at all levels and statistical quality control compliance rates. It can be connected wirelessly, the installation is simple and convenient, and the network is flexible; the monitoring station is preinstalled with the necessary software for the system, the nursing terminal has been embedded with the program software, and the equipment can be turned on after being powered on [11].

The medical IoTs can quickly assess patients and accurately classify patients. Based on the medical IoTs, the urinary real-time nursing model can effectively, quickly, and accurately obtain patient information and perform triage according to the criticality of the patient's disease. Through the IoTs system, it can transmit patient information to the doctor in real time so that the efficiency of patient consultation can be improved. In addition, the application of the medical IoTs to the urinary real-time nursing model can transmit patient information to rescue nurses in a timely manner so that the nurses can receive the information in time and carry out rescue operations in a timely manner. The medical IoTs is conducive to improving the work efficiency of nurses, and the application of the IoTs in the urinary real-time nursing model can significantly reduce the incidence of errors [12]. In addition, the intelligent identification of the medical IoTs can greatly reduce medication errors, avoid errors in patients' execution of medical orders, and significantly improve the quality of work. The medical IoTs provide transparent data through the communication layer and, at the same time, obtain the patient's physiological information through the perception layer. The nurse only collects the patient's vital signs and condition changes through the monitor and intelligent display screen, and at the same time transmits the patient's abnormal information to the doctor, which facilitates diagnosis and treatment, improves the patient's cure probability, and effectively protects the patient's life and health.

### 3.2. Model Software Design Based on Medical IoTs

The urinary real-time nursing model consists of two basic modules: a front-end application platform, a client, and a system data service center [13]. The front-end application platform receives various clinical information data related to the patient from the model data service middleware and saves data such as wards and basic patient information in the local database. At the same time, the data service middleware integrates the new data and interaction generated by the real-time nursing model of nursing information. Moreover, the data service center is also responsible for maintaining the consistency between the database and the nursing information urinary real-time nursing model and regularly obtaining and updating information from it (Figure 2). The entire nursing model exchanges various data through standard protocols, and through the cooperation of wireless smart mobile terminal equipment and software, it is possible for medical staff to query, input, modify, and save various data in real time in mobile locations and offices. Based on the change rules optimization algorithm, this method can not only reduce the number of shift nurses but also can reduce the ability level beyond the work level of nurses, help balance nurse workload, and improve the allocation efficiency of urinary nursing staff.

According to the characteristics of the algorithm, in addition to the general attributes, this nursing model also needs to add data acquisition time and coordinate information for positioning. The purpose of introducing coordinate information is to facilitate the conversion of a single data value into a data point in space, and its value is set to be equivalent to the obtained body data information. Any type of medical staff can log in and manage the urinary real-time nursing model through a browser on multiple platforms. According to different identities, the operations that the corresponding personnel can complete are also different. In urinary real-time nursing, the wireless sensor nodes attached to the patient can perceive the measurement values of multidimensional attributes, and the vector composed of the sensor measurement values of these multidimensional attributes represents the characteristic points of the patient's current physiological condition. The clustering algorithm can effectively find the abnormal points of the characteristic points, analyze and obtain similar data sets, and distinguish them from other data sets [14]. In the server data processing part, due to the environmental impact in the actual measurement, abnormal data will inevitably be generated. It is necessary to adopt a data analysis algorithm that conforms to medical reality and can eliminate abnormal data.

The realization of the medical IoTs is to bind intelligent sensing devices such as barcodes, sensors, and infrared sensors to urinary real-time nursing subjects, integrate them into various hospital information systems through network communication, and finally connect to the hospital's large-scale integration. The platform system realizes the functions of intelligent perception, data collection, remote monitoring, and information sharing of urinary real-time nursing subjects. The urinary real-time nursing model based on medical IoTs is applied to many aspects such as hospital staff management, item management, medical nursing, environmental monitoring, and information management, optimizing the urinary real-time nursing model and improving the overall efficiency of the hospital. The design and optimization of the urinary real-time nursing model based on medical IoTs is a process of gradual integration from shallow to deep. However, starting from the application of the IoTs intelligent system, it is gradually integrated on the basis of relevant protocols and standards and finally realizes a seamless network interconnection process between urinary real-time nursing and medical institutions, administrative management, and other related departments. Through horizontal comparison, the medical Internet can judge its position in the urinary real-time nursing model; through vertical comparison, it can judge and reflect the changes in the hospital's IoTs level in recent years.

## 4. Urinary Real-Time Nursing Model Optimization for Medical IoTs

### 4.1. Front-End Function Optimization of Urinary Real-Time Nursing

The optimized urinary real-time nursing model comprehensively observes the patient's life dynamics through horizontal and vertical forms. Urology is one of the important departments of the hospital. In recent years, in patients with urinary diseases, the traditional urinary nursing mode is low efficiency and has inconvenient problems, so we need to redesign and optimize urinary real-time nursing model, to improve the medical needs. Not only the overall monitoring content is more comprehensive, but the overall disease change content can be presented more clearly and intuitively. Doctors can better analyze the condition and make a diagnosis and treatment the first time. The optimized nursing urinary real-time nursing model comprehensively covers many aspects such as objective data, nursing observation, and nursing measures. Not only the recorded content is more prominent, but also more important points can be covered internally. In particular, it can effectively avoid errors caused by an incomplete handover and ensure the objectivity and integrity of nursing records afterward [15]. The optimization of real-time nursing mainly includes objective data, nursing observation, nursing measures, and other optimization, objective data streamlined, optimized; nursing observation more diverse, remote video, more humanized. The optimized urinary real-time nursing model is designed for the two main characteristics of medical IoTs and monitoring projects.  Figure 3 shows the front-end function optimization results of urinary real-time nursing based on the medical IoTs. Not only is the time for monitoring projects more flexible, but it can also take into account more monitoring projects. The time for nurses to record has been shortened to a large extent, and the workload for nurses to write has also been reduced. During the recording process, the nurses only need to simply fill in the relevant content in the urinary real-time nursing model, which simplifies the clerical work to the greatest extent and can avoid duplication of records to the greatest extent.

The optimized urinary real-time nursing model can make management goals clear, improve management efficiency, implement lean management, and improve the management level of the head nurse. The medical IoTs can apply the optimized design of the urinary real-time nursing model to carry out multifaceted, multiangle, and multilevel quality control of the ward nursing work and strengthen the quality control of the links. After optimization, the quality of ward management has been improved to varying degrees, and the quality of patient nursing has also been improved. Among them, public mandatory inspection items include pressure ulcer prevention and treatment, blood transfusion nursing, form nursing records, drug management, disinfection and isolation, hand hygiene, duty, shift system, and patients' identity recognition, checking of medical orders, execution of medical orders, management of rescue equipment, basic nursing satisfaction of high-quality nursing services, etc. The urinary real-time nursing model for medical IoTs includes inspection month, week, inspection date, bed number, result, the person in charge, focus problem or nurse, review date, and improvement effect. The urinary real-time nursing model can make detailed records of the problems in the examination and record the responsible persons; it can also rectify individual phenomena in time and enter the continuous quality improvement project for focused problems or nurses [16].

The monitoring and fault feature analysis of the urinary real-time nursing model need to be combined with the automatic detection of the urinary real-time nursing model. It realizes the feature analysis and detection of the urinary real-time nursing model through fault characteristic analysis and proposes the design and optimization method of the urinary real-time nursing model based on the IoTs technology. The medical IoTs use electrical metering chips to construct a fusion model of fault sample characteristic information for urinary real-time nursing. It realizes the reconstruction of the fault sample information of the urinary real-time nursing model in the operational amplifier and uses the open winding electric drive topology result to realize the fault monitoring and cluster analysis of the urinary real-time nursing model. It performs multidimensional feature fusion processing on the collected urinary real-time nursing information and extracts the high-order spectral characteristics of the urinary real-time nursing model. It realizes real-time monitoring of faults in the urinary real-time nursing model based on the distribution characteristics of the medical IoTs nodes. Finally, the hardware design of the urinary real-time nursing model is carried out, and the performance is verified through experimental tests, which demonstrates the superior performance of this method in improving the fault monitoring ability of the urinary real-time nursing model.

### 4.2. System Program Optimization of Urinary Real-Time Nursing

The data access layer is to perform operations such as adding, deleting, modifying, updating, and searching database data. When the system platform is running, a large amount of data is multiplexed, so the three-tier architecture will extract the commonly used data from each layer and perform data verification, cache processing, encryption, and decryption processing on the data for multiplexing in the three layers. Urinary real-time nursing system program optimization mainly includes data verification, cache processing, encryption decryption processing, uses the characteristics of bilinear, reduces the number of leaf nodes, and reduces the calculation involved in performance enhancement. In the medical IoTs, since the number of bilinear pairing operations and the length of the encryption key depend on the number of attributes in the table, the reduction of attributes will always reduce the calculations involved in providing performance enhancements.  Figure 4(a) gives the urinary nursing efficiencies of model hardware in their design and optimization. The number of random keys is always limited because it directly depends on the number of groups. IoTs devices, such as sensors, respiratory monitors, and other implantable medical devices, will continuously monitor the health of patients and send this information to the server. Since the number of bilinear pairs is proportional to the number of leaf nodes, the reduction in the number of leaf nodes is very advantageous.  Figure 4(b) shows the urinary nursing efficiencies of model software in their design and optimization. The urinary real-time nursing model enables the medical system to process the massive data generated by the IoTs devices to realize the monitoring and management of patients. Since the collected data is very sensitive and private health information, this model can ensure the confidentiality of data and the privacy of access.

The equipment management software has a complete role and authority management, which can intercept unauthorized requests, thereby effectively preventing authority overriding. The medical IoTs support multiple access operations such as mobile terminal applications, which can realize urinary real-time nursing status monitoring and intelligent management. The urinary real-time nursing model uses cloud computing technology to build a centralized management model of medical nursing, which has great advantages compared with the traditional decentralized and independent model [17]. The establishment of patient nursing files on the basis of the medical IoTs is to record all the health information of each patient. At the same time, the medical IoTs can also perform data mining on massive patient nursing files and statistically analyze the health status of patients. In order to more effectively protect and utilize data resources, the urinary real-time nursing model can adopt privacy protection technology based on inference control. The urinary real-time nursing model can set access rights and roles through the operating system and define the access rights of visitors; it can also use the network user identification system and a complete access control and authorization mechanism. The medical IoTs use encryption and other cryptographic technologies to ensure the authenticity of network user identities so that different roles can only access the information allowed by the security policy.

Due to diseases related to the urinary system, patients in urology surgery often have difficulty urinating and are less convenient to live independently. In addition to postoperative pain and postoperative physical inconvenience, patients are prone to bad moods during the entire treatment process. It is very helpful to improve the quality of nursing by humanizing the specific conditions of individual patients and discovering and alleviating patients' bad emotions in time [18]. The urinary real-time nursing model not only pays attention to the psychological nursing of patients but also pays attention to the nursing of patients in their lives during their hospitalization, giving them humane nursing, and avoiding the psychological resistance of patients due to hospital discomfort. At the same time, the urinary real-time nursing model has certain requirements for the nursing attitude of the nursing staff, ensuring that the nursing staff has a positive attitude, creating a good doctor-patient relationship, and creating a warm atmosphere for the treatment of patients. This is related to the staged detailed nursing before, during, and after the operation in the urinary real-time nursing model. Through the professional nursing of nursing staff, the patients will be guided on the precautions before and after the operation to avoid the patients from incorrect habits and practices.

## 5. Discussion

### 5.1. Hierarchical System Architecture of Urinary Real-Time Nursing Model

After the urinary real-time nursing model collects the basic information of the patient, all the data will be stored so that the doctors and nurses can view the data during the diagnosis and nursing process. The use of the medical IoTs can greatly improve the work efficiency of nursing staff and reduce errors, which can also comprehensively record the patient's physical characteristics. The same system response can also allow medical staff to directly observe the patient's physical changes and prevent some accidents. Workload statistics are mainly based on the use of medical IoTs technology, for the entire patient's various nursing content and treatment content are to carry out all information statistics and are to carry out grading component statistics for different nursing content [19]. As shown in Figure 5, the statistics will record the performance of the departments in accordance with various indicators and conditions to facilitate logistics statistics. The comprehensive application of medical IoTs technology to the infusion system has greatly improved the work efficiency of medical staff. The system can directly reflect the infusion information of each patient. Therefore, medical staff has more time to communicate with patients, and the corresponding problems can be handled more accurately through the system's response, which improves the quality of infusion nursing.

Figure 6(a)is the optimization factors of front-end function and systematic program in urinary real-time nursing model based on the medical IoTs. The urinary real-time nursing model is problem-centered, which has changed the problem that the previous nursing could not comprehensively and accurately assess the postoperative complications of patients. The medical IoTs can make timely judgments, notifications, and resolutions of patients' problems, and can find hidden dangers in time, take preventive measures in advance, and effectively reduce the incidence of postoperative complications, thereby effectively improving the quality of nursing and patient satisfaction.  Figure 6(b) shows the nursing satisfaction of front-end function and systematic program in urinary real-time nursing model based on the medical IoTs. With the implementation of the urinary real-time nursing model, the transition from terminal quality control to link quality control has been realized, and the dynamic management of the whole process of nursing work is truly achieved so that the management of nursing work will develop in a good direction. In the nursing training link, the medical IoTs have strengthened the ability of nursing staff to systematically identify, analyze, evaluate, and deal with problems that arise in different cases. The urinary real-time nursing model's training efforts to control risks within a reasonable range have further improved the quality of nursing, ensured patient safety, and made the learning and interactive atmosphere stronger. The urinary real-time nursing model further explains the problem-centered service concept and realizes the transformation of nursing work to the patient's all-round and full-course nursing.

The new urinary real-time nursing model adds a special medication recording area. By recording some special medications in the special medication area, the doctor can understand the patient's special medication more clearly. On the one hand, it can record the condition more comprehensively, and on the other hand, it can record some special conditions and conditions at any time and can better explain the special conditions later. Nursing does not need to record in the notebook when patrolling the ward and then return to the nursing station to input the information into the computer; nursing can be completed in real time by using a handheld mobile terminal and can complete nursing operations such as doctor order operations, blood sample collection, and vital signs entry. In the information management interface, all patient information is displayed in the form of a list, and the query button at the top can realize the query of the patient, supporting fuzzy and precise word queries. The user can click the Add button to jump to the patient registration page. The information is transmitted to the model layer to execute the update database function and then jump to the information management page.

### 5.2. Role Analysis of Medical IoTs in Urinary Real-Time Nursing Model

Through cluster application, grid technology, or distributed file system and other functions, the medical IoTs bring together a large number of different types of storage devices in the network through application software to work together to complete a system of data storage and business access functions. The urinary real-time nursing model does not use a certain storage device but a data-oriented service brought by the entire cloud storage system. The core of cloud storage is the combination of application software and storage devices, and the transformation from storage devices to storage services is realized through application software. The urinary real-time nursing model can automatically upload the body sign data collected by the medical instrument terminal; through the unified monitoring of the nursing doctor, it judges the excess sign data and communicates with the patient in time (Figure 7). The user can log in to the community medical service platform through the multifunction collector, directly make video calls with the doctor in charge, and consult the doctor about health, medication guidance, dietary advice, etc. For wired smart terminals, the communication device is connected to the wired network. The simple function transceiver only sends or receives one bit at a time, while the powerful one needs to pack the data, add the header, and encrypt and decrypt it with a secure encryption method.

All units connected to the bus in the urinary real-time nursing model have the ability to detect errors. Any unit on the bus will immediately notify other units on the bus after detecting an error, and the information sending unit that receives the error prompt will immediately force the end of the current sending and start to resend continuously until the sending is successful. The data layer includes data collection, modeling, and data storage. Data collection is to take out the patient's medical-related data from the database after the device is scanned and use data classification and modeling methods to store and manage the acquired business-related data in a unified manner. The database of the medical IoTs needs to have better server performance and a higher security database system to ensure data security. When the bedside of the ward control unit or the call button in the bathroom is pressed, the host at the nurse station will send out an audible and visual alarm signal, and the corridor display screen will display the bed number of the ward call at the same time, and the medical staff can go to the corresponding dealing with problems in the ward [20]. In order to reduce the impact of the ward alarm sound, a reset button can be installed at the nurse host to achieve the alarm elimination effect.

The urinary real-time nursing model plays a very important role as a bridge in the entire network; it also connects the network terminal and control processing and transmits data and control information. If the data of the network terminal part cannot be transmitted to the control processing, the basic functions of the mobile medical IoTs cannot be realized. If the data of the network terminal part cannot be fed back to the network terminal through the transmission network, the terminal cannot be effectively managed, and the advantages of the medical IoTs cannot be effectively utilized. The transmission network of the medical IoTs is the bridge of the entire medical IoTs system. What is transmitted in the network is the actual data collected by the network terminal and the control and processing result information that must be sent to the control. This constitutes the data flow of the medical IoTs, which is also medical IoTs attention. The medical IoTs middleware is the link between the urinary real-time nursing model reader and the information system, using standard protocols and interface technologies. In response to the different application service requirements of the medical IoTs, different medical IoTs middleware can be developed, such as medicine management middleware, medical equipment management middleware, personnel management middleware, electronic medical record transmission middleware, specimen management middleware, and material management middleware.

## 6. Conclusions

This paper conducts urinary real-time nursing model design based on medical IoTs, analyzes model hardware design based on medical IoTs, performs model software design based on medical IoTs, proposes the urinary real-time nursing model optimization based on medical IoTs, explores the front-end function optimization of the urinary real-time nursing, implements the system program optimization of the urinary real-time nursing, discusses the hierarchical architecture of the urinary real-time nursing model, and finally carries out the role function analysis of the medical IoTs in the urinary real-time nursing model. The urinary real-time nursing model plays a very important role as a bridge in the entire network; it also connects the network terminal and control processing and transmits data and control information. Through cluster application, grid technology, or distributed file system and other functions, the medical IoTs bring together a large number of different types of storage devices in the network through application software to work together to complete a system of data storage and business access functions. It performs multidimensional feature fusion processing on the collected urinary real-time nursing information and extracts the high-order spectral feature quantity of the urinary real-time nursing model. Since the number of bilinear pairing operations and the length of the encryption key depend on the number of attributes in the table, the reduction of attributes will always reduce the calculations involved in providing performance enhancements. The study results show that the urinary real-time nursing model based on medical IoTs can accurately and efficiently identify, manage, and integrate clinical nursing procedures and data such as patients, diagnoses, drugs, and can optimize nursing workflow, strengthen quality control, and improve nursing efficiency and provide patients with more convenient nursing services. The research results of this paper provide a reference for further research on the design and optimization of urinary real-time nursing models based on medical IoTs.

## Figures and Tables

**Figure 1:** Hardware design of urinary real-time nursing model based on the medical IoTs.

**Figure 2:** Software design of urinary real-time nursing model based on the medical IoTs.

**Figure 3:** Front-end function optimization results of urinary real-time nursing based on the medical IoTs.

**Figure 4:** Urinary nursing efficiencies of model hardware (a) and software (b) in their design and optimization.

**Figure 5:** Core electrical circuit of hierarchical system architecture in urinary real-time nursing model.

**Figure 6:** Optimization factors (a) and nursing satisfaction (b) of front-end function and systematic program in urinary real-time nursing model based on the medical IoTs.

**Figure 7:** Role analysis results of medical IoTs in the urinary real-time nursing model.

## Data Availability

No data were used to support this study.
